# Scanning Probe Microscopy Bone Marrow Determination of Steogenic Differentiation of Mesenchymal Stem Cells

This article has been retracted.

**DOI:** 10.1155/2022/6483087

**Published:** 2022-07-08

**Authors:** Xiandong Fu, Qixin Lian, Bo Zhang, Xinli Teng, Ying Chen, Yikun Qu, Zhuoxin Cheng, Linqi Guo

**Affiliations:** ^1^The First Affiliated Hospital of Jiamusi University, Department of General Surgery, Jiamusi 154000, China; ^2^The First Affiliated Hospital of Jiamusi University, Department of Tumour Surgery, Jiamusi 154000, China; ^3^Jiamusi University, Department of Pathophysiology, Jiamusi 154000, China; ^4^The Tumor Hospital of Jiamusi, Department of Tumor, Jiamusi 154000, China; ^5^The First Affiliated Hospital of Jiamusi University, Intensive Care Unit, Jiamusi 154000, China

## Abstract

To address the question of determining the osteogenic differentiation of mesenchymal stem cells, the bone marrow studies were performed using probe microscopy. All adherent bone marrow was used to isolate the bone marrow mesenchymal stem cells and expanded and purified in vitro. Its morphology under an inverted microscope was observed. We used Zuogui Pills to differentiate the separation methods. Alcian blue staining, modified calcium cobalt alkaline phosphatase staining, and neuron-specific enolase immunohistochemical staining were performed. The experimental results are shown below. The morphology of the isolated and purified cells was analyzed with an inverted microscope, and the isolated and purified cells were analyzed with Zuogui Pill. Alcian blue staining, modified calcium cobalt alkaline phosphatase staining, and neuron-specific enolase immunohistochemical staining confirmed that the cells differentiated into cartilage and osteoblasts, and the cell structure and morphology were similar to those of the bone marrow mesenchymal stem cells. The results showed that the adherent mode of cells obtained from the whole bone marrow was the rat bone marrow mesenchymal stem cells, and the Zuogui Pills could induce multidirectional differences in the bone marrow mesenchymal stem cells.

## 1. Introduction

Most of the methods used to treat bone defects include severe damage to the free space and deep grafts in the grafted area. In recent years, bone tissue engineering has opened up a broad field of vision for the treatment of various types of bone defects. Testis is one of the three major components of the bone marrow engineering, and selecting the appropriate testis is an important part of bone marrow engineering. Bone marrow mesenchymal stem cells refer to nonhematopoietic stem cells in the bone matrix that can differentiate into osteoblasts capable of necessary induction. However, the osteogenic function of mesenchymal stem cells is weak and the ossification process is slow. Therefore, the question of how to improve the osteogenic potential of MSCs to be effective on osteoblasts may be an important link in the process of bone marrow transplantation. According to the Chinese herbal medicine “Kidney governs the bone,” Chinese herbal medicine was used in Guiban to invigorate the kidney to study the osteogenic properties of MSCs, as shown in Figure 1.

## 2. Literature Review

A large number of experiments have shown that bone remodeling is a new discipline with a wide variety of disciplines. It uses the principles of biology, medicine, and tissue engineering to treat the damaged bones or treat bone diseases. Bone defect is a global health problem, and its treatment faces serious challenges. Bone defects are usually caused by injury or physiological bone resorption. Bone deformity due to trauma is a medical problem in craniofacial and orthopaedic surgery. Bone reconstruction is required to treat the defect and to improve the patient's quality of life. In addition to injury, bone remodeling can also be considered in some bone diseases caused by gender, age, and infection, such as bone loss, disease-induced bone and tooth loss [1].

Ajay states that the nonhematopoietic stem cells in the bone marrow are mesenchymal stem cells (MSCs), and the bone-received “fibroblasts” promote the healing of many tissues, including the nasal periphery [2]. Mesenchymal stem cells are stem cells with the ability to self-regenerate and differentiate. In the early 1970s, Fatih etal. recognized the possible presence of unrestricted fibroblasts in mouse bone [3]. Sergeev's understanding of MSCs is mainly based on the properties of stem cells cultured in vitro, such as the ability to reproduce indefinitely, multiply, and differentiate in vitro [4]. Later, Criman et al. it found that MSCs X are not only derived from bone marrow but also exist in other tissues such as fat, umbilical cord blood, amniotic fluid, placenta, dental pulp, synovium, and muscle bonds [5].

According to the current study, a probe-based microscopy method is used for bone marrow research. Bone marrow mesenchymal stem cells (BMSCS) are the cells that are easily expanded and have many different characteristics. Under differential induction, MSCs can differentiate into osteoblasts, chondroblasts, myoblasts, adipocytes, and stromal cells [6]. In recent years, it has been observed that the occurrence and development of MSCs are similar to those of the bone marrow. The failure of MSCs to differentiate into osteoblasts or to improve the differentiation of adipocytes is one of the reasons for bone loss. Most of the methods used to treat bone defects involve severe damage to the graft and gravity of the graft. However, in recent years, bone marrow engineering has opened up the prospect of treating a variety of bone defects [7]. Testis is one of the three major components of the bone marrow engineering, and selecting the appropriate testis is an important part of the bone marrow engineering. Bone marrow mesenchymal stem cells refer to the nonhematopoietic stem cells in the bone matrix that can differentiate into osteoblasts capable of necessary induction. However, the osteogenic function of the mesenchymal stem cells is weak and the ossification process is slow. Therefore, the question of how to improve the osteogenic potential of the MSCs to be effective on osteoblasts may be an important link in the process of bone marrow transplantation.

## 3. Discussion and Research

### 3.1. Research Status Quo

Stem cells are the cells that are able to regenerate themselves permanently or over an extended period of time and change over at least one generation. Several biologists have used various methods to create human embryonic stem cells which are capable of permanent and totipotent growth. Stem cells have limited or delayed self-regeneration and many different potentials in vitro, making it possible to grow many human cells, even tissue noses and organs in the lab. According to the differentiation of stem cells, stem cells can be divided into three categories: totipotent stem cells, pluripotent stem cells, and specialized stem cells. TSCs can vary in many cells, and theoretically in individuals. The most representative of TSC is ESC. PSCs have different capabilities for different cells, but cannot be modified to be independent. For example, hematopoietic stem cells can differentiate in different cells but not in other cells. Under appropriate conditions, BMSCs can differentiate into cells such as bone, bone, fat, muscle, muscle, nerve-like cells, cardiomyocytes, and stromal cells that support hematopoietic stem cells. MSC stem cells can only differentiate into one or two similar cells, such as neural stem cells that can differentiate into neurons and glia. As in normal growth biology, cellular differentiation is stable and often irreversible. Cells differ in one direction and do not return to their original position. For example, hematopoietic stem cells can only differentiate into RBC, WBC, PLT, etc. but not differentiate into other types of cells [8].

### 3.2. Purpose and Significance of the Research

Stem cells have limits on the length or duration of self-regeneration and vary widely. They are the foundation of tissue care and tissue repair. Due to these characteristics of stem cells, it has become a new way to treat certain diseases, which has been widely used in medicine: hematopoietic stem cell transplantation for vascular diseases and limbal stem cell transplantation for ophthalmic diseases. Stem cell transplants are often used to treat children with cerebral palsy and diabetes. Spinal cord injury is a problem related to the spine. The theory has always been that neurons cannot regenerate after injury, which is a common problem among orthopedic surgeons. With the discovery of stem cells, stem cells can theoretically be differentiated into genes and cultures in human tissues or in vitro tissues, with the potential to mutate and treat traumatic neuronal diseases such as the spinal cord injury [9].

In recent years, Chinese scientists have also carried out research on the use of stem cell conversion therapy to treat spinal cord injuries and have achieved positive results. Based on the above research, some scientists have used stem cell therapy to treat neurological diseases with positive results. According to the theory of traditional Chinese medicine, “the kidney strengthens the soul, regulates the tendons, and strengthens the tendons.” The bone marrow is the extraordinary home, consisting of two parts, the spinal cord and the marrow of the cerebrum and midbrain [10]. As a traditional treatment method, the method of invigorating the kidney and nourishing the spirit has a therapeutic effect on the spine. In view of the above situation, this study aimed to differentiate BMSCs into neuron-like cells by applying Chinese herbal medicine to invigorate the kidney in vitro, and to provide an experimental basis for Chinese herbal compound invigorating the kidney and prescribing psychotropic drugs for the treatment of SCI [11] as shown in Figure 2.

### 3.3. Clinical Application Value

Spinal cord injury is a common clinical disease. Some scholars have found that about 10%–20% of the spinal cord injury occurs to varying degrees after a spinal fracture. About 40% of the spinal cord injuries will occur in cervical spine fracture and dislocation and about 10%–20% of the spinal cord injury will occur in thoracic and lumbar vertebrae. At the same time, the incidence of spinal cord injury rises by about 12000 cases every year. The consequences of spinal cord injury are disastrous including the patients' movement and sensation disorders. The treatment of spinal cord injury in modern medicine has not yet shown exciting therapeutic effects and the patients are accompanied by lifelong drugs and rehabilitation training. Most of the patients with spinal cord injury cannot recover their functional and sensory impairment, which affects the individual spirit and thoughts of the patients and causes a serious burden on the family and society. The current difficulty in the treatment of the spinal cord injury is the motivation for further research [12].

According to the theory of traditional Chinese medicine, the experimental research on spinal cord injury with single or compound Chinese medicines mainly focuses on regulating qi and promoting the blood circulation. The commonly used Chinese medicines include astragalus membranaceus, salvia miltiorrhiza, panax notoginseng, safflower, and red peony root, etc. Traditional medical treatment for patients with spinal cord injury mainly focuses on promoting blood circulation, improving local microcirculation, alleviating local spinal cord tissue edema, inhibiting free radicals and alleviating lipid peroxidation in order to partially repair spinal cord injury. According to the traditional theory of “The kidney stores spirit and generates marrow.” the traditional Chinese medicine for tonifying kidney and filling spirit should have a certain effect on the treatment of the spinal cord injury. Through the review of the literature, it is found that there are few experimental researches and clinical reports on the treatment of spinal cord injury by using traditional Chinese medicine for tonifying kidney. The purpose of this research is to induce the differentiation of BMSC into neuron-like cells by using the traditional Chinese medicine tonifying kidney filling spirit to provide experimental basis for the experimental research and clinical treatment of spinal cord injury in the future and a new idea for the later related researches [13].

Modern studies have shown that BMSC has the ability to transform into neuron-like cells and DMEM combined with dithiyl ethanol (BME), fetal bovine serum, or DMEM combined with basic fibroblast growth factor (bFGF) are usually used to induce BMSC to differentiate into neuron-like tissues [6]. There are few experimental researches on the differentiation of BMSC into neuron-like cells in vitro induced by the traditional Chinese medicine or compound Chinese medicine. On this basis, guided by traditional Chinese medicine theory, this paper attempts to induce differentiation of BMSC in vitro by compound Chinese medicine of tonifying kidney and filling spirit. Compound traditional Chinese medicine has control characteristics of many active ingredient, multiple targets , and multiple links. Limited in the present study condition, the mechanism of Chinese traditional medicine cannot be explained very clearly. The scholars' understandings are also different. Through the experiment, it is hoped that stem cell theory provides a new train of thought and method and also provides some experimental basis for traditional Chinese medicine theory [14].

### 3.4. Classification of Stem Cells

In daily life, there are many animals that can grow the same limbs as the original through their own repair mechasims. This phenomenon is widespread in nature, such as salamander, octopus, and leech. This phenomenon in nature is attributed to the existence of “stem cells” in the animal, allowing it to repair itself after an injury through differentiation of stem cells and allowing missing limbs to be rebuilt. The name of stem cells comes from the English word stem cell. Stem in English means “trunk” or “origin,” which means stem cells have the characteristics like trunk that can grow branches, leaves, blossom, and bear fruit on the trunk [15]. The meaning is not easy to understand. Stem cells do not differentiate and develop; they can produce a variety of cancer cells and tissues and play an important role in the growth and development of cancer cells in the body. According to its different stages, it can be divided into embryonic stem cells and adult stem cells. According to their different abilities, they can be divided into totipotent stem cells, pluripotent stem cells, and specialized stem cells [16].

## 4. Experiment and Research

### 4.1. Isolation and Culture of Rat Bone Marrow Mesenchymal Stem Cells (BMSC)

Mice were sacrificed by removing the throat and immersed in 75% ethanol for 10 minutes. The bilateral femurs of the aseptic rats were excised, the soft tissue was excised, and the epiphysis was excised together with the epiphyseal plate. We used a 5 ml syringe to draw Dmem-hg medium to flush the femoral cavity. It was then filled with rinse solution and was rinsed 3 times. The aqueous solution was reconstituted and mixed, centrifuged in a centrifuge (1000 rpm, 5 min), filled with supernatant, washed twice with dMEM-HG medium, and centrifuged again to collect cells. In this experiment, double DMEM-Hg-resistant medium containing 10% FBS (to remove contaminants) was used as the medium, which was placed in a 25 mL culture flask, under room temperature CO2, 37°C, 5% CO_2_-saturated humidity incubator. The medium was changed after 72 hours and then after every 72 hours. When the cells reached 85% of the bottom of the flask, the culture medium was discarded, and 0.25% trypsin was preheated at 37°C for 10 min to further digest the culture. Due to the good adhesion properties of BMSCs, nonadherent heterologous cells can be removed by liquid exchange and these cells grew well during the culture process [17].

### 4.2. “Zuogui Pill” Induced Differentiation of Rat Bone Marrow Mesenchymal Stem Cells (BMSC)

Three passages of MSCs were digested with 0.25% trypsin and cut with 10% FBS. At a cell density of 2 × 10° cells/mL, the MSCs were seeded into eight 6-well plates with 24 × 24 mm lids, 1 mL wells. After 48 hours, when the cell plate reached 70%, a 6-well plate was used to divide it into a control group. One 6-well plate for each of the groups I, II, III, IV, V, VI, and VII. The plate was supplemented with 3 ml of DMEM-HG medium containing 10% FBS per well. The counting solution was added to each well in the study group, except for the DMEM-HG containing an average of 10% FBS. The final concentration was 2.0 mg/ml. The culture medium was changed every 72 hours. After a total of 14 days of induction and mutation, the experiment was completed [18].

### 4.3. Morphological Observation of BMSC

Gi EMSA staining and inverted microscope were used to observe the growth morphology of the BMSC, the performance of adherent growth, the morphological changes after fluid exchange and passage, the growth rate, and the growth form, and other cell morphologies.

### 4.4. Cell Morphology Observation under Microscope

Gi EMSA staining and inverted microscope were used to observe the growth morphology of the induced BMSC, the performance of adherent growth, the morphological changes after fluid exchange and passage, the growth rate, the growth form, and other cell morphologies [19].

### 4.5. Isolation of BMSC in Rats

The mesenchymal stem cells were widely found in mesenchymal derived tissues, such as fat tissue, blood, bone marrow, and muscle. Bone marrow was currently recognized by scholars as the tissue with the largest amount of mesenchymal stem cells. The BMSC accounted for 1/1000-1/100000 of bone marrow nucleated cells, and the bone marrow had become the most commonly used material for the isolation of mesenchymal stem cells. The amount of BMSC in vivo was very small, so it was necessary to isolate, purify, and amplify BMSC in vitro to obtain sufficient amount of BMSC for tissue engineering and experimental researches in vivo and in vitro. Currently, the commonly used methods included the whole bone marrow adherent method, the density gradient centrifugation method, the immunomagnetic bead method, and the flow cytometry isolation method [20]. Although, a variety of methods could be used to isolate the BMSCS from the bone marrow, there was currently no optimal method and different methods had different problems. For the imunomagnetic bead method, if the magnetic bead was larger than the mechanical extrusion of the cell, the cell would cause relatively large damage, affecting the cell activity. Generally, the negative isolation method was used for the immunomagnetic bead method. Even if the magnetic bead was combined with the useless cells, relatively pure BMSC could be obtained. Because the amount of BMSC in the body was small, it required more magnetic beads and would cost a lot to use this method [21]. Flow cytometry used laser light to irradiate the cells to produce specific fluorescence for collection, which may damage the cell itself and affect its cell activity. At the same time, there was no specific marker for BMSC at present, so the immunomagnetic bead method and the flow cytometry sorting method were not widely applied [22]. In the current researches, the whole bone marrow adherent method and the density gradient centrifugation method were more applied, or the combination of the two methods was used. Density gradient centrifugation could effectively isolate the red blood cells, white blood cells, monocytes, and so on, and had little effect on the cellularity. However, it destroyed the cytokines and the adhesion-promoting substances that were favorable for the growth of BMSC in the microenvironment, which might have adverse effects on the expansion of BMSC in vitro. Whole bone marrow adherent isolation of BMSC was based on the characteristics of the adherent growth of the BMSC and the characteristics of the suspended growth of the blood cells. After multiple fluid changes, unadherent blood cells were removed to obtain relatively pure BMSC [23]. Although this method took a long time and the cell components obtained were complex, various components such as trophoblast cells and some cytokines were retained in the bone marrow solution and was washed with the medium, which can promote the growth and expansion of the BMSC [24].

### 4.6. Test Results

After the primary cells were cultured for 72 h and the solution was changed, the adherent part of the BMSC was observed under an inverted microscope. Most of them were polygonal and short spindle in shape and the nuclei were round or oval. After 1 week, the cells grew in colony form, and after 12 days, the cells were able to cover the bottom of the bottle. After passage, the BMSC was round, and it began to grow adherent 24 h later. The BMSC recovered the adherent growth performance and the cells gradually extended to grow into long spindle shape and aggregated into clusters. About 14 days later, the cells filled up 85% of the flask bottom and the cell culture was be carried out. After passage, the growth rate of the cells was significantly accelerated, which could be passed once a week. Most of the cells were fibroblast-like cells with relatively consistent morphology, which initially showed colony growth and then gradually fused into slices. In this experiment, the third generation of the BMSC was used for induction and differentiation. Based on the above reasons, the isolated, purified, and amplified cells were BMSC'90, which was disproved according to the characteristic of the multidirectional differentiation of the BMSC. From the experimental results, the DMEM/F12 medium without traditional Chinese medicine was added to the control group to induce the cells of the third generation and no positive cell expression of the ALP, AB, and NSE was detected by histochemistry and immunohistochemistry staining, indicating that there was no differentiation of osteoblasts, chondrocytes, and neuron-like cells. Thc Zuogui Pill group was used to induce differentiation of cells passing it to the third generation. The experimental results showed that there were a large number of positive cell expressions of the ALP, AB, and NSE, which proved that the cells obtained by whole bone marrow adherence method in the experiment were BMSC.

## 5. Conclusion

According to the theory of traditional Chinese medicine and from the academic viewpoint of “The kidney controls bone and generates marrow,” the experiment confirmed that the whole prescription of Zuogui Pill could induce the differentiation of rat BMSC into osteoblasts, chondrocytes, and neuron-like cells, which also proved that the physiological function of BMSC and spirit stored in kidney was similar. Experimental results also proved Zuogui Pill as an inducer of BMSC differentiation was not directional differentiation and there were a number of different direction of differentiation, which may be related to the fact that the traditional Chinese medicine composition was complicated. And there were different medicinal ingredients in each component of the TCM compound and each component contained various medicinal ingredients in the process of drug preparation, which can make a difference in chemical reaction. The compatibility law of traditional Chinese medicine is based on the guidance of the theory of traditional Chinese medicine. Chinese compound is the best representative of the compatibility law of traditional Chinese medicine and also is the best way to reflect the academic thoughts of traditional Chinese medicine. On the basis of clarifying the multidirectional differentiation induction effect of Zuogui Pill on the rat BMSC, the drug withdrawal research was used to observe the results of the influence of various components of Zuogui Pill on the induced differentiation of BMSC into neuron sample cells. And the drugs with a stronger induction effect on the differentiation of BMSC into neuron sample cells could be sorted out for the benefit of future research or medical practice.

## Figures and Tables

**Figure 1:** Differentiation of the bone marrow mesenchymal stem cells.

**Figure 2:** Types of stem cell transplantation.

## Data Availability

The data used to support the findings of this study are available from the corresponding author upon request.
